This article has been retracted.

# Rural Workplace Sustainable Development of Smart Rural Governance Workplace Platform for Efficient Enterprise Performances

**DOI:** 10.1155/2022/1588638

**Published:** 2022-06-03

**Authors:** Yingli Wu, Wanying Ma

**Affiliations:** ^1^Agricultural and Rural Development Institute, Heilongjiang Provincial Academy of Social Sciences, Harbin, China; ^2^Changchun Guanghua University, College of Business, Jilin, Changchun 130033, China

## Abstract

In the long developmental process, China's agriculture has transformed from organic agriculture to inorganic agriculture. New technologies have made the modernization of agriculture possible. However, most older people who are engaged in agriculture may not completely understand the modernization of agriculture. Based on the limitations of traditional image target detection methods, a deep learning-based pest target detection and recognition method is proposed from a blockchain perspective, to analyze and research agricultural data supervision and governance and explore the effectiveness of deep learning methods in crop pest detection and recognition. The comparative analysis demonstrates that the average precision (AP) of GA-CPN-LAR (global activation-characteristic pyramid network-local activation region) increases by 4.2% compared with other methods. Whether under the Inception or ResNet-50 backbone networks, the AP of GA-CPN-LAR is significantly better than other methods. Compared with the ResNet-50 backbone network, GA-CPN-LAR has higher accuracy and recall rates under Inception. Precision-recall curve measurement shows that the proposed method can significantly reduce the false detection rate and missed detection rate. The GA-CPN-LAR model proposed here has a higher AP value on the MPD dataset than the other target detection methods, which can be increased by 4.2%. Besides, the accuracy and recall of the GA-CPN-LAR method corresponding to two representative pests under the initial feature extractor are higher than the MPD dataset baseline. In addition, the research results of the MPD dataset and AgriPest dataset also show that the pest target detection method based on convolutional neural networks (CNNs) has a good presentation effect and can significantly reduce false detection and missed detection. Moreover, the pest regulation based on blockchain and deep learning comprehensively considers global and local feature extraction and pattern recognition, which positively impacts the conscientization of agricultural data processing and promotes the sustainable development of rural areas.

## 1. Introduction

In the long-term development process, Chinese agriculture has transformed from organic agriculture to inorganic agriculture. New technologies make it possible to modernize agriculture. However, most older adults working in agriculture may not fully understand the modernization of agriculture. Currently, there are fewer Internet services for agricultural technology and agricultural knowledge. The breadth of geography makes it difficult to achieve the target technology. Therefore, it is very urgent to analyze and study agricultural modernization from the perspective of information technology. Agriculture should develop in the direction of science and intelligence, which is also crucial for the development of smart agriculture [1, 2]. In addition, in recent years, blockchain technology has developed rapidly, which is one of the ten typical technology applications of the Internet. The blockchain is a digital record updated and distributed in chronological order with encryption protection. Compared with a linear blockchain, the blockchain stores information in each block, connects them to each other, and shares the entire network among all participants. It has the characteristics of openness and autonomy, which are extensively applied in increasing fields and industries. This technology is also a means and tool to serve economic activities to facilitate the development of related transactions [3–5]. The depth of deep learning is compared to shallow machine learning methods, which is the current research hotspot in the field of machine learning. It is a general term for learning methods based on deep learning networks originating from artificial neural networks. The deep learning network started in the 1940s and mainly solved various machine problems by trying to simulate the cognitive mechanism of the human brain.

Agriculture is China's primary industry, and its integration with blockchain started late in China. There is no doubt that the integration of blockchain and agriculture is very necessary with the rapid development of big data technology and modern technology. Lin et al. analyzed the role of blockchain technology in improving the efficiency of sustainable agricultural development. They proposed an e-agriculture model system with blockchain infrastructure [6]. Au emphasized the application value of blockchain technology in agriculture, IoT, energy, and finance [7]. Khan et al. took secure IoT blockchain data as the research object and proposed a hybrid model based on recurrent neural networks by using deep learning algorithms to analyze the agriculture and food industries. They evaluated the performance under different numbers of households, providing a reference for supply chain practitioners to develop advanced deep learning forecasting policies using the latest technology [8]. To sum up, some research results have been achieved in the application of blockchain technology in the agricultural field. However, there are still few studies exploring the combination of blockchain and deep learning methods in the agricultural field.

In this context, this work proposes an image target detection method that combines global and local features to find a detection method suitable for pest identification and build an intelligent agricultural data supervision platform. Besides, this scheme's feasibility in agricultural data supervision is analyzed to provide a reference for sustainable agricultural development.  Figure 1 displays the organizational structure of this article.

## 2. Methods

### 2.1. The Blockchain Technology

It is an intelligent peer-to-peer network. Blockchain can identify and disseminate information through distributed databases [9, 10]. The blockchain ecosystem is developed based on Bitcoin. With the continuous improvement and optimization of algorithms, blockchain has been gradually integrated with different industries. The formation of scalable smart contracts in this process makes the integration of the sharing economy possible, and industrialization can be accomplished. Smart contracts are one of the key elements for mainstream blockchain platforms. This is actually a computer program based on which information can be processed and stored. According to its definition, the blockchain consists of data blocks, and different data blocks correspond to different network transaction information. These blocks can verify the validity of the data information, from which the next block is generated [11]. In general, blockchain is a distributed accounting method under decentralization. Its principal function is to enable different objects participating in it to establish technical trust. The development and maturity of this technology have attracted many parties. The application of this technology in the agricultural field is also very concerned [12]. In essence, blockchain is a value transfer trust protocol and a database under decentralization. This feature of decentralization also makes the technology very secure. Based on the background of agricultural modernization, blockchain is introduced to construct the rural intelligent data supervision and government platform considering that data supervision is important for the intellectual development of agriculture.

In addition, the application of blockchain technology to the sustainable development of rural areas has many advantages, as shown in Figure 2.

It can be found from Figure 2 that the advantages of blockchain technology in the sustainable development of rural areas are mainly reflected in four aspects: decentralization, openness, independence, and security. Decentralization means that blockchain technology does not rely on additional third-party rural management agencies or hardware facilities, and there is no central control. Except for the self-contained blockchain itself, each node realizes information self-verification, delivery, and management through distributed accounting and storage. In addition to the encrypted private information of transaction parties, the blockchain's data are open to all local people in rural areas. Anyone can query the blockchain data and develop related applications through the open interface, so the information of the entire rural system is highly transparent. Independence means that the entire blockchain system does not rely on other third parties, and all nodes can automatically and securely verify and exchange data within the system without any human intervention. Security indicates that attackers cannot arbitrarily manipulate and modify the network data as long as they cannot control 51% of all data nodes, which makes the blockchain safe and avoids artificial data changes in rural areas.

Figure 3 reveals the operating principle of blockchain technology.

### 2.2. Deep Learning and Convolutional Neural Network

Deep learning promotes the development of artificial intelligence technology. Under deep learning, the system can learn relevant features actively. The elementary idea of deep learning is to express the input information hierarchically by learning large quantities of samples and stacking feature hierarchies [13, 14]. This method imitates the cognition and behaviors of human brains. The deep learning-based neural networks can understand data information of images and texts from shallow to deep, from simple to complex, and from concrete to abstract. The entire construction of attributes and characteristics is also a process of seeking the law of data development. The theoretical model of deep learning is presented in Figure 4.

Among the components of the deep learning method, convolutional neural network (CNN) is a type of feedforward neural network. It applies to the processing of data formed by a grid structure [15, 16]. In image processing, CNN can extract and process data features. The core structure of CNN includes the convolutional layer, the pooling layer, the normalization layer, and the fully connected layer. Among them, the convolutional layer is a unique component of CNN [17], and its operational implementation can be expressed as follows:

(1) $$\begin{array}{c} y\left(t\right)=\int x\left(a\right)k\left(t-a\right)\text{da}, \end{array}$$

where *x* represents the input vector, *k* represents the convolution kernel, and *t* represents different moments of the corresponding convolution operation. Among the convolutional layers, the convolution kernel is the most critical component, and the output corresponding to the convolution can be obtained by the convolution kernel through uniform sliding at the moment of dimension. Convolution operations involving multiple dimensions can be expressed as`:

(2) $$\begin{array}{c} Y\left(i,j\right)=\sum_{m}\sum_{n}X\left(m,n\right)K\left(i-m,j-n\right), \end{array}$$

where *X* represents the two-dimensional input matrix, and *K* represents the two-dimensional convolution kernel. The convolutional layer in CNN can reduce the calculation parameters and the amount of calculation significantly.

The major function of the pooling layer is to reduce the dimensionality of the feature map, which can reduce the number of parameters and retain the initial feature information of the image to the greatest extent as well [18]. The convolution operation is a linear operation method with limitations in processing and expressing nonlinear data. Hence, a nonlinear activation function is introduced into the CNN structure to achieve the nonlinear modeling of neural networks [19]. In addition, this activation function can also filter redundant information so that the data features can be retained. The essence of the normalization layer in CNN is the zero-average processing for the convolutional layer structure in the neural network. For images, it is the normalization processing operation for each channel. The nonlinearity of the corresponding data can be reduced through normalization. During network training, the overall direction of network learning is determined by the loss function, and the correctness of the training process is also inseparable from the loss function. The excellent performance of CNN in many fields is due to these special network composition structures.

CNN has an excellent performance in feature extraction. In the deep learning field, there have been many CNN-based target detection algorithms. In recent years, target detection technology has developed rapidly. However, in the agricultural field, the recognition and detection of crop pests have not yet achieved practical deep learning applications. Traditional pest recognition methods mainly depend on the manual design of features. The feature descriptors involved are color, shape, and texture. Although this method can identify pests, the basis of manual design is not universal. The design of feature descriptors needs to be based on different types of pests and their specific images. The breakthrough of deep learning in image recognition and detection provides possibilities for image target detection. The primary process of pest recognition in the agricultural field includes feature extraction and pattern recognition. Unlike traditional methods, the deep learning method uses CNN for feature extraction. The image target detection based on the deep learning method also shows good performance in pattern recognition. The excellent characteristics of this method in image target detection are also applicable in crop pest recognition and detection. The deep learning method provides a new direction for the detection and recognition of pests. However, there are still some problems in practical applications. In most cases, the feature extractor chooses the backbone network. Nevertheless, due to the serious problem of target occlusion in the virtual image environment, the adaptability of the network for feature extraction is poor. In addition, due to the small size of pests themselves, neural network algorithms, such as Faster Region-CNN (R-CNN), are not effective in detecting small targets. Regardless of this problem, a pest recognition and detection method that integrates global and local features is proposed based on CNN. Given the small-sized detection target, a top-down feature transfer structure is introduced to improve the effective detection of small targets. A global activation-characteristic pyramid network (GA-CPN) is introduced to solve the problem of severe occlusion in pest target detection, achieving the high-quality detection and recognition of pests.

### 2.3. Design and Establishment of GA-CPN and LAR Models

#### 2.3.1. Design of GA-CPN

LAR includes the channel attention and spatial attention modules. When designing this module, a global pooling operation *F*_*gp*_ is introduced in the CNN model, which is specifically expressed as:

(3) $$\begin{array}{c} z_{p}=F_{gp}\left(x_{c}\right)=\frac{1}{H_{g}\times W_{g}}\sum_{i=1}^{H_{g}}\sum_{j=1}^{W_{g}}x_{c}\left(i,j\right), \end{array}$$

where *x*_*c*_ represents the branch tensor of the module, *H*_*g*_ × *W*_*g*_ represents the channel size of the feature map, and *z*_*p*_ represents the pooling output of the corresponding feature map. Introducing *F*_*gp*_ aims to remove the function of the feature map on the feature weights *H*_*g*_ and *W*_*g*_. This operation can remove the effect brought by the spatial information by placing the three-dimensional feature map on a one-dimensional vector. In the meantime, *z*_*p*_ corresponding to each channel can describe the corresponding feature map composition information. On this basis, a two-layer fully connected CNN is introduced to implement feature extraction *U*_*c*_ of *z*_*p*_, which is specifically expressed as:

(4) $$\begin{array}{c} U_{c}=\sigma_{2}\left(P_{2}^{T}\sigma_{1}\left(P_{1}^{T}Z_{p}+b_{1}\right)+b_{2}\right), \end{array}$$

where *P*_1_ represents the learning parameter of the first fully connected layer, *P*_2_ is the learning parameter of the second fully connected layer, and *b*_1_ and *b*_2_ correspond to the bias.

The rectified linear unit (ReLU) is taken as the activation function of the first layer and sigmoid as the activation function of the second layer. The input global feature map corresponding to *X*_*g*_ and the output activation vector corresponding to *U*_*c*_ are subjected to weighted average processing, which is specifically expressed as follows:

(5) $$\begin{array}{c} \tilde{x_{c}}=x_{c}\cdot u_{c}, \end{array}$$

where *x*_*c*_ represents the characteristic activation maps corresponding to different channels.

The main purpose of designing the spatial attention module is to note the small size detection target position and remove some influences brought by the channel information as well. This module is trained based on supervised learning. First, for the removal of each channel information, a global convolution operation *F*_*gc*_ is introduced in this module design, which is expressed as follows:

(6) $$\begin{array}{c} z_{s}\left(i,j\right)=F_{gc}\left(X_{g}\right)=\sum_{c=1}^{C_{g}}\sum_{m}\sum_{n}X_{g}\left(i+m,j+n,c\right)K\left(m,n,c\right)+b, \end{array}$$

where *K* represents the convolution kernel corresponding to the operation, its size is *m* × *n* × *C*_*g*_, and *b* represents the bias. In the global convolution process, the number corresponding to *K* is 1, the size of the corresponding output feature map is *H*_*g*_ × *W*_*g*_ × 1, and the number of corresponding channels is 1. At this time, the features at different positions correspond to the spatial features of the image. On this basis, two sets of dilated convolutions with different convolution kernel sizes are used for learning and activating the matrix so that the spatial receptive field can be expanded, which is specifically expressed as follows:

(7) $$\begin{array}{c} U_{s}=\sigma_{2}\left(K_{2}*\sigma_{1}\left(K_{1}*Z_{S}+b_{1}\right)+b_{2}\right), \end{array}$$

where *K*_1_ and *K*_2_ represent the convolution kernel, and *b*_1_ and *b*_2_ represent the bias. In this module, ReLU and sigmoid are also selected as activation functions. In the network training, the pixel set-based cross-entropy loss PCE is introduced as the loss function, which is specifically expressed as follows:

(8) $$\begin{array}{c} PCE\left(U_{S},U_{gt}\right)=\frac{1}{H_{g}\times W_{g}}\sum_{i=1}^{H_{g}}\sum_{j=1}^{W_{g}}-U_{gt}\left(i,j\right)\log\;U_{s}\left(i,j\right), \end{array}$$

where *U*_*gt*_ represents the activation map formed at the labeled bounding box, and *U*_*S*_ represents the spatial feature activation matrix. The relevant target information is preserved in the form of exponential operation at each channel to preserve the global information of the feature map. A spatial activation global feature map *X*_*g*_ based on the spatial dimension is finally obtained by stacking the activation feature maps on each channel.

#### 2.3.2. Local Activation Region (LAR) module

In the deep learning field, R-CNN has good performance in extracting and expressing local image features, which can classify and detect various images [20, 21]. The network is generated based on the LAR to optimize the performance of R-CNN in image processing. LAR mainly includes two modules: contextual feature enhancement and self-attention activation [22, 23]. The former aims to solve the problem of insufficient target information of small size [24, 25]. For the candidate frames in the standard region generative network, based on Rol pooling, local feature *X*_l_ can be extracted from all the candidate frames obtained by training from the global activation feature map *X*_*g*_. The specific expression is as follows:

(9) $$\begin{array}{c} X_{l}\left(i,j,c\right)=\frac{k^{2}}{wh}\sum_{m=x_{1}}^{wkli}\sum_{n=y_{1}}^{hkli}\tilde{X_{g}}\left(m,n,c\right), \end{array}$$

where *k* represents the size of the output feature map, which takes seven under normal circumstances. The average pooling operation is performed on the cropped subregions obtained by Rol pooling, and finally, the local feature map corresponding to the candidate frame can be output [26, 27]. In this module, the candidate frames in different directions are expanded to contain more contextual information. The quality of the pest information contained in the final local feature map is higher based on this module [28, 29].

The self-attention activation module aims to buffer the insensitivity of the fully connected neural network in the spatial information [30, 31]. The module includes three parallel convolution operations. The local feature maps' output by the three branches can be expressed as follows:

(10) $$\begin{array}{c} f\left(X_{l}^{\prime }\right)=K_{f}*X_{l}^{\prime },\\ g\left(X_{l}^{\prime }\right)=K_{g}*X_{l}^{\prime },\\ h\left(X_{l}^{\prime }\right)=K_{h}*X_{l}^{\prime }, \end{array}$$

where *K*_*f*_, *K*_*g*_, and *K*_*h*_ represent the convolution kernels, and the corresponding size is 1 × 1 × *C*_l_. Based on these three branches, the corresponding feature map can contain the feature information of each position, thereby completing the interactive processing of the information. The corresponding output *s* can be expressed as:

(11) $$\begin{array}{c} s=f{\left(X_{l}^{\prime }\right)}^{T}g\left(X_{l}^{\prime }\right). \end{array}$$

Furthermore, the dimensionality is reduced through convolution operation, and the softmax activation function is used to learn the weight value at each position. Specifically, the activation matrix is expressed as:

(12) $$\begin{array}{c} U_{a}\left(i,j\right)=\frac{\exp\left(s\left(i,j\right)\right)}{\sum_{m=1}^{k}\sum_{n=1}^{k}\exp\left(s\left(m,n\right)\right)}. \end{array}$$

Under such a training method, the self-attention activation matrix obtained above is merged with the third network branch structure so that the local position information can be noted.

The image target detection method based on the two modules of GA-CPN and LAR is introduced to design and construct the agricultural data supervision and governance model, in an effort to provide a direction for sustainable development in rural areas [32]. The image target detection method that combines the two modules of GA-CPN and LAR is denoted as GA-CPN-LAR.

### 2.4. Construction of the Agricultural Data Supervision Model

With the continuous development and advancement of agricultural science and technology, the number of data resources has also increased rapidly. However, due to the influence of hierarchical and decentralized factors, fragmented data make the accurate acquisition of data difficult, which has affected the development of agriculture towards science and intelligence [33]. Hence, it is very necessary to find a method suitable for integrating and processing complex agricultural data. A scientific system for agricultural data supervision and governance should follow the principles of truth-seeking, systematicity, timeliness, accuracy, and predictability. From the demand perspective, the scientific supervision of agricultural data and the establishment of the government platform should comprehensively consider factors such as data collection, data organization, data storage, and data sharing [34]. The implementation or smooth progress of this process requires the blessing of data fusion or algorithms. Data workers serving the platform should try their best to participate in the various processes of data processing. Yan et al. [35] quoted blockchain technology and deep learning technology into the dataset and classified it after integrating a large amount of complex data. They found that combining these two technologies has broad applicability, and the data classification processing accuracy is high [35]. The agricultural data supervision and governance model constructed from a blockchain perspective is shown in Figure 5. Among them, the analytical focus is pest detection and recognition, which is implemented through deep learning methods [36–39].

As can be seen from Figure 5, the implementation of agricultural data supervision requires blockchain technology. First, a detailed design of the agricultural supervision and governance plan is carried out. Then, data development, data collection, and data analysis are performed on the set platform. Finally, the effective data are stored in the cloud network disk to use and disseminate the data at any time and integrate new experimental data [40]. For the GA-CPN-LAR target detection method, armyworm (A), corn borer (CB), plant louse (PL), wheat spiders (WS), bollworm (B), and *Mamestra brassicae* Linnaeus (MB) are selected as the research objects [41, 42]. Under the MPD and AgriPest datasets, several target detection methods, namely single-shot multi-box detector (SSD), are used. A single-shot multi-box detector is an object detection algorithm to produce a fixed-size set of bounding boxes and scores of object class instances present in these bounding boxes, followed by a non-maximum suppression step to produce the final detection. SSD consists of two parts: the backbone and the head. The backbone model is usually a pretrained image classification network. The SSD head is one or more convolutional layers added to the backbone. The output is interpreted as the bounding box and category of objects in the spatial location of the last layer of activation. The feature pyramid network (FPN) is a feature extractor designed to improve accuracy and speed. It replaces the feature extractor in detectors such as Faster R-CNN and generates a higher quality feature map pyramid. An FPN consists of bottom-up and top-down paths. The bottom-up path is a commonly used convolutional network for feature extraction. Spatial resolution decreases from bottom to top. The semantic value of each layer increases as higher-level structures are detected. The Faster R-CNN can be simply regarded as an upgraded version of R-CNN and Fast R-CNN or a system of “Regional Generation Network + Fast R-CNN,” which replaces the selective search method in Fast R-CNN with the regional generation network. The AP (average precision) value and precision-recall curve are used as evaluation indicators for the comparison between the above methods and the proposed GA-CPN-LAR.

## 3. Results and Discussion

### 3.1. Image Target Detection Based on MPD Dataset

Figure 6 compares SSD, FPN, and Faster R-CNN target detection methods with the GA-CPN-LAR model proposed here on the MPD dataset.

The distribution and change of AP value in Figure 6 suggest that the GA-CPN-LAR model has a higher AP value than the other target detection methods, which is increased by 4.2%. The AP value of each detection method under different CNN backbone networks shows a similar trend. Specifically, the AP value of the SSD method is 51.35. Under the initial backbone network, the AP value of Faster R-CNN is 66.73, and that of FPN is 70.03. In contrast, the AP value of the GA-CPN-LAR model is 71.97. Under the ResNet-50 backbone network, the AP value of the Faster R-CNN, FPN, and GA-CPN-LAR is 70.97, 78.14, and 80.75, respectively. Therefore, the AP value of several target detection methods in the initial state can be increased by 2.1% compared with ResNet-50.

Two crop pests, corn borer and bollworm, are taken as examples. Under the Inception backbone network, the precision-recall curves of several target detection methods under the MPD dataset are shown in Figures 7(a) and 7(b).

Data changes in Figure 7 suggest that compared with the baseline of the MPD dataset, the accuracy and recall rate of the GA-CPN-LAR method corresponding to the two representative pests under the Inception feature extractor are higher.

The reason is that the proposed target detection method introduces the unique structure of the characteristic pyramid. The proposed GA-CPN-LAR can locate the crop pest target for each multilevel feature map so that the pests can be located more accurately. Introducing global activation features can improve the extraction quality of image features effectively. Introducing a contextual attention mechanism can learn local activation matrices, making the neural network more sensitive to the exact positions of the pests in different regions. This is also the reason for the improvement in the overall detection performance of GA-CPN-LAR proposed in the case of local features. The precision-recall curves show that the GA-CPN-LAR method can reduce the probability of false detection and missed detection for pest detection effectively.

### 3.2. Image Target Detection Based on AgriPest Dataset

Under the AgriPest dataset, the target detection methods of SSD, FPN, and Faster R-CNN are compared with the proposed GA-CPN-LAR. The results are shown in Figure 8.

Under the AgriPest dataset, the Faster R-CNN target detection method performs unsatisfactorily in detecting pests. In contrast, the proposed GA-CPN-LAR deep target detection method has a better AP value than other target detection methods, which can be increased by 3.2–9.8%.

In addition, two crop pests, corn borer and bollworm, are taken as examples. Under the Inception backbone network, the precision-recall curves of several target detection methods under the AgriPest dataset are shown in Figures 9(a) and 9(b).

Compared with other target detection methods, the proposed GA-CPN-LAR method has higher accuracy and recall rate. Its overall changing law shows similar changes and distributions to the MPD dataset.

The results under the MPD dataset and the AgriPest dataset suggest that the proposed CNN-based pest target detection method has a good presentation effect and can significantly reduce the false detections and missed detections, pointing out a good direction recognizing and detecting crop pests in the field environment. Besides, the method has a high detection accuracy. The above results reveal that the deep learning-based pest detection GA-CPN-LAR method applies to the agricultural data supervision and governance platform.

### 3.3. Implementation of the Agricultural Data Supervision and Governance Platform

From the blockchain perspective, the GA-CPN-LAR pest target detection method based on deep learning is introduced into the platform. The implementation of the agricultural data supervision and governance platform is shown in Figure 10.

This blockchain-based data supervision platform essentially includes the data layer, neural network detection layer, consensus layer, and application layer. Among them, the neural network detection layer is the core. In the process of agricultural modernization and intellectualization, the agricultural data supervision and management platform is vital for the identification and detection of pests. The pest and disease supervision based on blockchain and deep learning comprehensively considers global and local feature extraction and pattern recognition, which has a positive impact on promoting the scientization of agricultural data processing and promoting the sustainable development of rural areas. Obviously, blockchain technology and deep learning have great application potential in agricultural data analysis and governance.

## 4. Conclusions

This work introduces deep learning methods for the design and implementation of agricultural data supervision and governance platforms based on the effectiveness of blockchain technology in network transmission to promote the long-term sustainable development of rural areas. The GA-CPN-LAR pest detection method is put forward. The main conclusions are as follows: (1) With the MPD dataset, GA-CPN-LAR has a higher AP value than other target detection methods, increasing by 4.2%. (2) Compared with the baseline of the MPD dataset, the GA-CPN-LAR method corresponding to two representative pests under the initial feature extractor has higher precision and recall. (3) Under the AgriPest dataset, the Fast R-CNN object detection method performs poorly in detecting pests. In contrast, the AP value of the proposed GA-CPN-LAR deep object detection method outperforms other object detection methods by 3.2%∼9.8%. In addition, the results of the MPD and AgriPest datasets show that the CNN-based pest and disease target detection method reported here has a good presentation effect, significantly reducing false detection and missed detection. Therefore, it points out a good direction for identifying and detecting crop pests and diseases in the field environment. Furthermore, the regulation of pests and diseases based on blockchain and deep learning comprehensively considers global and local feature extraction and pattern recognition, which positively impacts the scientization of agricultural data processing and even promotes the sustainable development of rural areas. Therefore, the research results can provide a feasible method for the intelligent and scientific development of agricultural governance.

The agricultural data supervision and governance platform is a very complicated system. However, only pest detection and recognition are analyzed due to the influences of different objective factors. In addition, the size of the selected detection samples is small. Hence, the research samples will be increased to discuss more aspects of agricultural data supervision in future works.

## Figures and Tables

**Figure 1:** Text organization.

**Figure 2:** Advantages of blockchain technology in rural sustainable development.

**Figure 3:** How blockchain technology works.

**Figure 4:** Deep learning model.

**Figure 5:** The agricultural data supervision and governance model.

**Figure 6:** Comparison of several target detection methods' AP values under MPD dataset.

**Figure 7:** Precision-recall curves based on Inception under MPD dataset: (a) corn borer and (b) bollworm.

**Figure 8:** Comparison of several target detection methods' AP values under the AgriPest dataset (A denotes armyworm, CB denotes corn borer, PL denotes plant lice, WS denotes wheat spider, B denotes cotton bollworm, MB denotes brassica, and mAP denotes average accuracy).

**Figure 9:** Precision-recall curve based on Inception under the AgriPest dataset: (a) corn borer and (b) bollworm.

**Figure 10:** Implementation of the agricultural data supervision and governance platform.

## Data Availability

The simulation experiment data used to support the findings of this study are available from the corresponding author upon request.
